The article "Rapid Identification of the Multiple Absorbed Bioactive Components and Metabolites in Rat Serum after Oral Administration of Wu-Jia Sheng-Hua Capsule by UPLC-ESI-MS" was published in 2013. Journal: J Anal Methods Chem.

# Rapid Identification of the Multiple Absorbed Bioactive Components and Metabolites in Rat Serum after Oral Administration of Wu-Jia Sheng-Hua Capsule by UPLC-ESI-MS

**DOI:** 10.1155/2013/318961

**Published:** 2013-05-14

**Authors:** Fang Geng, Fashan Wang, Taobo Zou, Kuiyuan Zhu, Wei Ma, Guanghui Tan, Ning Zhang

**Affiliations:** ^1^School of Chemistry & Chemical Engineering, Harbin Normal University, Shi Da Nan Road, Harbin 150025, China; ^2^Duo Duo Pharmaceutical Co. LTD., An Qing Street, Jiamusi 154000, China; ^3^College of Jiamusi, Heilongjiang University of Chinese Medicine, Guang Hua Road, Jiamusi 154000, China

## Abstract

To identify the compounds absorbed in rat serum after the oral administration of Wu-Jia Sheng-Hua (WJSH) capsule, a traditional Chinese medicine (TCM) compound prescription, an ultraperformance liquid chromatography coupled with electrospray ionization mass spectrometry (UPLC/ESI-MS) method, was established. The chromatographic separation of the absorbed compounds and metabolites was achieved with an ACQUITY UPLC BEH C18 column (2.1 mm × 50 mm, 1.7 *μ*m) under a gradient elution. The mobile phase was composed of acetonitrile and water buffered with ammonium acetate (10 mM) and formic acid (0.1%, V/V). Twelve absorbed compounds and four metabolites were found. Seven of the absorbed compounds were identified by ESI-MS. The identification of absorbed compounds might be helpful for the better understanding of the mechanisms underlying the pharmacological effects of WJSH capsule.

## 1. Introduction

Chinese postpartum care (Zuoyuezi) has been regarded as a crucial rite-to-passage for the woman's recovery and the transition to motherhood after childbirth [1]. The use of Sheng-Hua-Tang, a well-known traditional Chinese medicine (TCM) compound prescription, during the postpartum has been popular in Chinese communities over a long period. Previous study has shown that Sheng-Hua-Tang use during the first month of the postpartum period may have a positive effect on women's health-related quality of life, especially in terms of role limitations due to physical health and emotional problems [2]. Wu-Jia Sheng-Hua capsule (comprising *Radix et Caulis Acanthopanacis Senticosi*, *Radix Angelicae Sinensis*, *Rhizoma Chuanxiong*, *Semen Persicae*, *Radix Glycyrrhizae*, and *Rhizoma Zingiberis Preparata*), derived from Sheng-Hua-Tang, has been used widely in Chinese women to promote blood flow, resolve blood stasis, ease postchildbirth pain, reduce bleeding volume and shorten bleeding duration after induced abortion in Chinese women [3, 4]. The material base, namely the bioactive components, of Wu-Jia Sheng-Hua (WJSH) capsule is still unclear, though the prostaglandin F2alpha (PGF_2*α*_), prostaglandin E2 (PGE_2_), endothelin (ET), and nitrogen monoxide (NO) levels were found to be partially responsible for the curative effects and recovery benefits of WJSH capsule on induced abortion with vaginal haemorrhage [4].

The article "Rapid Identification of the Multiple Absorbed Bioactive Components and Metabolites in Rat Serum after Oral Administration of Wu-Jia Sheng-Hua Capsule by UPLC-ESI-MS" was published in 2013. Journal: J Anal Methods Chem.

TCM serum pharmacochemistry, based on hypothesis that active compounds should appear in blood after administration of TCM, was proposed by Homma et al. [5, 6]. In the past two decades, it was proved to be helpful in recognizing the real active components in TCM and in gaining a better understanding of the mechanisms under the therapeutic effects of TCM [7–9].

In the present study, an ultraperformance liquid chromatography coupled with electrospray ionization mass spectrometry (UPLC/ESI-MS) method was developed and applied for investigating the serum pharmacochemistry of WJSH capsule. It was thought that TCM expresses its effects through multicomponents with multitargets [10]. The identification of WJSH's multiple absorbed bioactive components and metabolites might be helpful for better understanding the mechanisms under its therapeutic effects.

## 2. Experimental Method 

### 2.1. Reagents and Chemicals

 Syringin, protocatechuic acid, liguiritin, ferulic acid, isofraxidine, chlorogenic acid, and liqustilide (standards) were purchased from National Institute of Control of Pharmaceutical and Biological Products (Beijing, China).

Acetonitrile, methanol, formic acid, and ammonium formate (HPLC grade) were obtained from Merck (Darmstadt, Germany) and Sigma-Aldrich (St. Louis, MO, USA), respectively. Other chemicals are of analytical grade.

Wu-Jia-Sheng-Hua capsule and each single herb in the prescription of Wu Jia Sheng Hua capsule were gifts from Duo Duo Pharmaceutical Co. LTD. (Heilongjiang, China). 

### 2.2. UPLC Conditions

The chromatographic separation of the absorbed components and metabolites were performed on a Waters ACQUITY UPLC system (Waters Corp., Milford, MA, USA) equipped with an UV detector, an autosampler, an ACQUITY UPLC BEH C18 column (2.1 × 50 mm, 1.7 *μ*m), and an automatic thermostatic column oven. The mobile phase consisted of (A) water buffered with ammonium acetate (10 mM) and formic acid (0.1%, V/V) and (B) acetonitrile. The column temperature was kept at 40°C. The elution of the target compounds was conducted in a gradient mode with the volume percentage of B changed from 5% to 50% in the initial 10 minutes and from 50% to 80% in the next 6 minutes. The flow rate was 0.4 mL/min, and the injection volume was 8 *μ*L. 

### 2.3. MS Conditions

 To obtain the MS and MS/MS data of the investigated compounds, a Waters Quattro Premiere XE triple-quadrupole mass spectrometer (Micromass MS Technologies) was coupled to the abovementioned UPLC system. Ionization was performed in the positive electrospray (ESI) mode. The mass range was set at *m/z* 100–1000 Da with the scan time being 0.5 s. The ionization parameters were as follows: interval time, 0.2 s; capillary voltage, 3.5 kV; cone voltage, 35 kV; ionization resource temperature, 120°C; desolvation temperature, 380°C, desolvation gas flow rate, 500 L/h (N_2_); and cone gas flow rate, 50 L/h (N_2_). MassLynx software (version 4.1) and QuanLynx software were used for system control and data processing, respectively.

The article "Rapid Identification of the Multiple Absorbed Bioactive Components and Metabolites in Rat Serum after Oral Administration of Wu-Jia Sheng-Hua Capsule by UPLC-ESI-MS" was published in 2013. Journal: J Anal Methods Chem.

### 2.4. Sample Preparation

 5 mL methanol was added to 1 mL blank rat serum sample or WJSH capsule serum sample. The mixture was vortexed for 3 min. and centrifuged for 15 min. (4°C, 5000 rpm). 5 mL supernatant was dried under gentle nitrogen gas stream at 37°C. The residues were kept at −20°C. Before analysis, each residue was reconstituted in 1 mL methanol and centrifuged for 15 min. (4°C, 14,000 rpm). 8 *μ*L supernatant was injected for UPLC-ESI-MS analysis.

### 2.5. Serum Pharmacochemistry Study of WJSH Capsule

The extracts of WJSH capsule and raw medicinal materials of WJSH capsule were prepared separately. 10 mL methanol was added to 0.4 g WJSH or each raw medicinal material. The suspensions were sonicated for 30 min., centrifuged (3000 rpm) for 15 min., and filtered through 0.45 *μ*m micropore film (Millipore, USA). The supernatants were collected as extracts.

Male Sprague-Dawley rats (230 g ± 10 g, Experimental Animal Center of Heilongjiang University of Traditional Chinese Medicine) were randomly divided into eight groups (six for each): Group A to Group H. All care and handling of animals were performed with the approval of Institutional Authority for Laboratory Animal Care of Heilongjiang University of Traditional Chinese Medicine. 

After 12 hours of fasting, normal saline (blank control) and extract of WJSH capsule were given intragastrically to rats in Group A and Group B, separately. Extracts of raw medicinal materials were given intragastrically to rats of the other 6 groups (one extract per group). The dosage was 1.5 mL/100 g body weight, and the administration frequency was once daily in three consecutive days in each group. At forty minutes after the last administration, 5 mL blood was collected *via* hepatic portal vein. The blood samples were centrifugated for 10 min. at 5000 rpm at 4°C to separate serum samples. The residues were kept at −20°C until analysis. 

## 3. Results and Discussions

### 3.1. Optimization of UPLC-ESI-MS Conditions

To purify the serum sample, the protein precipitation, liquid-liquid extraction, and solid-phase extraction methods were tried. Finally, the simple protein precipitation method with methanol was chosen, since most investigated compounds were found in the purified samples.

The article "Rapid Identification of the Multiple Absorbed Bioactive Components and Metabolites in Rat Serum after Oral Administration of Wu-Jia Sheng-Hua Capsule by UPLC-ESI-MS" was published in 2013. Journal: J Anal Methods Chem.

As compared to methanol-water system, higher resolution, better peak shape, and faster elution of compounds were achieved using acetonitrile-water system buffered with ammonium acetate and formic acid. Therefore, this system was used as mobile phase. The chromatographic separation of the absorbed components and metabolites was conducted in gradient elution mode to overall reduce the retention time of these compounds characterized by different polarities. The timetable of gradient elution was listed in Table 1.

For the ESI-MS conditions, the stronger responses of all compounds were obtained in positive ionization mode than in negative mode. Thus, positive mode was employed in the total ion current (TIC) chromatograms of WJSH capsule serum samples in the *m/z* range of 100 to 1000 Da. 

### 3.2. Identification of Absorbed Components

 The multiple bioactive components in TCM could be simultaneously identified using the UPLC-ESI-MS technique. It is generally helpful in better understanding the mechanisms underlying TCM's therapeutic effects. 

The serum pharmacochemistry study of WJSH capsule was conducted in rats orally administered with WJSH Capsule. Then, the absorbed bioactive components including their metabolites were identified by the established UPLC-ESI/MS method. The typical TIC chromatograms of WJSH capsule extract, WJSH capsule serum sample, and blank serum sample were shown in Figure 1. Twelve chemicals of which chromatographic peaks appeared in the TIC chromatograms of WJSH capsule serum sample and WJSH capsule extract, but not in that of the blank serum sample, were presumed to be the absorbed components. Similarly, four chemicals whose chromatographic peaks presented only in the TIC chromatograms of WJSH capsule serum sample, but not in that of the WJSH capsule extract or the blank serum sample, were supposed to be metabolites. 

By comparing the MS/MS spectra, the chromatographic peaks in TIC chromatogram of WJSH capsule serum sample versus the standards, respectively, seven absorbed components were identified unequivocally. For instance, the MS/MS spectrum of peak 5 was compared with that of the isofraxidine standard. These MS/MS spectra were shown in Figure 2. Since the quasi-molecular ion at *m/z* 223 [M + H]^+^, fragmentation ions at *m/z* 192 [M + H-OCH_3_]^+^, and at *m/z* 161 [M + H-OCH_3_-OCH_3_]^+^ were found simultaneously in the MS/MS spectra of peak 5 and the standard of isofraxidine; this absorbed component was confirmed to be isofraxidine. The other six components were identified in the same way. The chemical structures of the identified components were shown in Figure 3. The other five absorbed components and the four metabolites were not identified and need further investigation.

The article "Rapid Identification of the Multiple Absorbed Bioactive Components and Metabolites in Rat Serum after Oral Administration of Wu-Jia Sheng-Hua Capsule by UPLC-ESI-MS" was published in 2013. Journal: J Anal Methods Chem.

By comparing the TIC chromatograms of serum samples, WJSH capsule, WJSH capsule without *Radix et Caulis Acanthopanacis Senticosi,* and *Radix et Caulis Acanthopanacis Senticosi* alone, isofraxidine was confirmed to be originated from *Radix et Caulis Acanthopanacis Senticosi*. Similarly, the original plant(s) of the other absorbed components and metabolites were confirmed. These TIC chromatograms were shown in Figure 4. The retention times, MS/MS data, and original plants of the absorbed components and metabolites were listed in Tables 2 and 3, respectively. 

By revealing the bioactive components of TCM compound prescriptions, serum pharmacochemistry studies might be significantly helpful in better understanding the mechanisms under the therapeutic effects of these prescriptions. For instance, WJSH capsule and Danggui-Shaoyao-San have been used extensively in Chinese women to enhance uterine involution after giving birth and alleviate dysmenorrhea, respectively [11, 12]. In pharmacological experiments, the prostaglandins (PG) levels regulation was proved to be partially responsible for the myometrium contraction stimulation and inhibition effects of WJSH capsule and Danggui-Shaoyao-San, separately [4, 12]. In previous and present serum pharmacochemistry investigations, identical (ferulic acid and liqustilide) and different (syringin, protocatechuic acid, liguiritin, isofraxidine, and chlorogenic acid for WJSH capsule; paeoniflorin sulfonate, albiflorin, paeoniflorin, butylidenephthalide, and senkyunolide I for Danggui-Shaoyao-San) bioactive components in WJSH capsule and Danggui-Shaoyao-San were identified [13]. By conducting comparative pharmacokinetic and pharmacological experiments, the major bioactive components in WJSH capsule and Danggui-Shaoyao-San related to the up- and downregulation effect on myometrium contraction might be confirmed, and the influence of other coexisting components on these effected might be revealed. Thus, the mechanisms under WJSH capsule and Danggui-Shaoyao-San's therapeutic effects might be elucidated.

## 4. Conclusion

In this study, an UPLC-ESI-MS method was established for investigating the serum pharmacochemistry of WJSH capsule. In this way, twelve absorbed bioactive components and four metabolites were found in rat serum. Seven of the absorbed bioactive components were identified. These results might be helpful for better understanding the mechanisms underlying the therapeutic effects of WJSH capsule.

The article "Rapid Identification of the Multiple Absorbed Bioactive Components and Metabolites in Rat Serum after Oral Administration of Wu-Jia Sheng-Hua Capsule by UPLC-ESI-MS" was published in 2013. Journal: J Anal Methods Chem.

## Figures and Tables

**Figure 1:** Total ion chromatogram of (a) WJSH capsule extract, (b) mixture of standards, (c) WJSH capsule serum sample, and (d) blank rat serum in positive mode. Peaks: 1, syringin; 2, protocatechuic acid; 3, liguiritin; 4, ferulic acid; 5, isofraxidin; 6, chlorogenic acid; 7, liqustilide; M1, M2, M3, and M4, stand for metabolites 1, 2, 3 and 4, respectively.

**Figure 2:** MS/MS spectra of (a) peak 5 in TIC chromatogram of WJSH capsule serum sample; (b) standard of isofraxidine.

**Figure 3:** Identified bioactive components of WJSH capsule absorbed into rat plasma after oral administration.

**Figure 4:** TIC chromatograms of serum samples: (a) WJSH capsule; (b) *Radix et Caulis Acanthopanacis Senticosi* alone; (c) WJSH capsule without *Radix et Caulis Acanthopanacis Senticosi*. Peaks: 1, syringin; 2, protocatechuic acid; 3, liguiritin; 4, ferulic acid; 5, isofraxidine; 6, chlorogenic acid; 7, liqustilide; M1, M2, M3, and M4 stand for metabolites 1, 2, 3, and 4, respectively.

**Table 1:** The timetable of gradient elution in UPLC conditions.

Time (min.)	Solvent A (%, V/V)	Solvent B (%, V/V)
Initial	95	5
10	50	50
16	20	80

Solvent A: water buffered with ammonium acetate (10 mM) and formic acid. Solvent B: acetonitrile.

**Table 2:** The retention times, +ESI-MS/MS data (*m/z*), and origins of the absorbed components in rat serum after oral administration of WJSH capsule.

No.	Rt (min.) extract/plasma	Positive ions (*m/z*)	Origins	Identification
1	2.05/2.04	395 [M + Na]^+^, 373 [M + H]^+^	*Radix *et* Caulis Acanthopanacis Senticosi *	Syringing
2	2.71/2.73	155 [M + H]^+^, 137 [M + H-H_2_O]^+^, 111 [M + H-CO_2_]^+^	*Radix *et* Caulis Acanthopanacis Senticosi*, *Radix Glycyrrhizae,* *Rhizoma Chuanxiong,* *Rhizoma Zingiberis Preparata *	Protocatechuic acid
3	3.25/3.28	419 [M + H]^+^, 441 [M + Na]^+^, 403 [M-CH_3_]^+^	*Radix Glycyrrhizae *	Liquiritin
4	3.43/3.40	195 [M + H]^+^, 180 [M + H-CH_3_]^+^, 151 [M + H-CO_2_]^+^,	*Radix *et* Caulis Acanthopanacis Senticosi*, *Radix Angelicae Sinensis,* *Rhizoma Chuanxiong,* *Radix Glycyrrhizae *	Ferulic acid
5	3.89/3.91	223 [M + H]^+^, 192 [M + H-OCH_3_]^+^, 161 [M + H-OCH_3_-OCH_3_]^+^	*Radix *et* Caulis Acanthopanacis Senticosi *	Isofraxidine
6	4.22/4.27	355 [M + H]^+^, 377 [M + Na]^+^, 193 [M-C_9_H_7_O_3_]^+^, 181 [M-C_7_H_11_O_5_]^+^, 175 [M-C_9_H_7_O_3_-H_2_O]^+^	*Radix *et* Caulis Acanthopanacis Senticosi*, *Radix Glycyrrhizae *	Chlorogenic acid
7	4.44/4.46	191 [M + H]^+^, 175, 151, 137	*Radix Angelicae Sinensis *	Liqustilide
8	4.73/4.69	223, 205, 195	*Radix Angelicae Sinensis* *Semen Persicae *	—
9	5.10/5.13	237, 222	*Radix *et* Caulis Acanthopanacis Senticosi *	—
10	10.87/10.89	247, 232	*Radix *et* Caulis Acanthopanacis Senticosi *	—
11		194, 176	*Radix Glycyrrhizae *	—
12	13.30/13.27	431, 388, 370	*Rhizoma Chuanxiong *	—

The article "Rapid Identification of the Multiple Absorbed Bioactive Components and Metabolites in Rat Serum after Oral Administration of Wu-Jia Sheng-Hua Capsule by UPLC-ESI-MS" was published in 2013. Journal: J Anal Methods Chem.

**Table 3:** The retention times, +ESI-MS/MS data (*m*/*z*), and origins of the metabolites in rat serum after oral administration of WJSH capsule.

Peak no.	Rt (min.) extract/plasma	Positive ions (*m/z*)	Origin
M1	4.78/4.79	207, 229	*Radix Angelicae Sinensis* *Rhizoma Chuanxiong * *Semen Persicae *
M2	5.12/5.14	262, 244	*Radix *et* Caulis Acanthopanacis Santicosi *
M3	6.94/6.92	189, 154	*Radix Angelicae Sinensis* *Rhizoma Chuanxiong * *Semen Persicae *
M4	7.59/7.61	323, 245, 308	*Rhizoma Zingiberis Preparata *
